# The Regulation and Characterization of Mitochondrial-Derived Methylmalonic Acid in Mitochondrial Dysfunction and Oxidative Stress: From Basic Research to Clinical Practice

**DOI:** 10.1155/2022/7043883

**Published:** 2022-05-24

**Authors:** Yige Liu, Shanjie Wang, Xiaoyuan Zhang, Hengxuan Cai, Jinxin Liu, Shaohong Fang, Bo Yu

**Affiliations:** ^1^Department of Cardiology, Second Affiliated Hospital of Harbin Medical University, Harbin, China; ^2^The Key Laboratory of Myocardial Ischemia, Chinese Ministry of Education, 246 Xuefu Road, Nangang District, 150086 Harbin, China

## Abstract

Methylmalonic acid (MMA) can act as a diagnosis of hereditary methylmalonic acidemia and assess the status of vitamin B12. Moreover, as a new potential biomarker, it has been widely reported to be associated with the progression and prognosis of chronic diseases such as cardiovascular events, renal insufficiency, cognitive impairment, and cancer. MMA accumulation may cause oxidative stress and impair mitochondrial function, disrupt cellular energy metabolism, and trigger cell death. This review primarily focuses on the mechanisms and epidemiology or progression in the clinical study on MMA.

## 1. Introduction

MMA is an intermediate metabolite in the catabolism of four amino acids (i.e., isoleucine, threonine, methionine, and valine) as well as odd-chain fatty acids. MMA can be used to diagnose hereditary methylmalonic acidemia and as a first-line functional indicator of subclinical vitamin B12 deficiency [1]. And existing cross-sectional studies suggest that MMA is considered a potential risk factor for cardiovascular events. Although plasma levels of MMA exceed the universal reference interval with age, other factors may be involved in major organs. In epidemiological studies, MMA is related to the risk and poor prognosis of numerous chronic diseases. It is largely evidenced that MMA has a significant relationship to chronic diseases (e.g., aging, diabetes, obesity, and kidney dysfunction) [2, 3]. In particular, MMA is a mitochondrial toxin that can disrupt redox homeostasis by inhibiting electron transport complex II [4]. With the increase in concentrations of MMA, mitochondrial energy metabolism can be altered. Thus, disorders of mitochondrial energy metabolism can promote free radicals to be generated intracellularly, which damages mitochondrial DNA [5]. Furthermore, MMA is suggested to be a biomarker of oxidative stress conditions [6]. As a promising novel biomarker, MMA may optimize the risk stratification of diseases and provide a potential target for the study of disease mechanisms.

## 2. Circulating MMA in Clinical Diagnosis

### 2.1. MMA and Vitamin B12 Deficiency

The relationship between MMA and vitamin B12 (vitamin B12, Cb1) deficiency dates to the 1960s [7, 8]. Some medical institutions consider the MMA assay a more appropriate response to vitamin B12 activity than the conventional vitamin B12 test. Still, MMA testing has not been widely used, and there is no consensus on its clinical use. MMA is one of the indicators of Cb1 deficiency. Vitamin B12 deficiency refers to a prevalent condition attributed to nutritional deficiency and the damage of vitamin B12 function. It affects the synthesis of leukocytes and red blood cells, usually manifesting as megaloblastic anemia and neurological disorders [7]. This can be attributed to a defective Cb1 modification or transport step, which decreases the activation efficiency of methylmalonyl-CoA mutase (MCM) and methionine-lyase (MS), further leading to the accumulation of MMA and homocysteine (Hcy) in vivo [8, 9]. Accordingly, both constitute accurate biomarkers of vitamin nutritional and functional deficiencies of vitamin B12 (Cb1) [8]. It has been proposed that oxidative stress disorder can lead to the inactivation of Cb1 oxidative metabolism [6]. As a result, older, cardiovascular disease, renal insufficiency, or cancer patients exhibit higher susceptibility to “functional vitamin B12 deficiency” [10–12], which is characterized mainly by elevated MMA and Hcy levels, but normal Cb1 levels. In general, many studies have shown that Hcy is positively correlated with the severity of coronary heart disease, is a key risk factor for the cardiovascular system, and is a good predictor of disease assessment in coronary heart disease [13]. However, there is also evidence that Cb1 is a highly bound protein, and the concentration of free Cb1 is difficult to measure while circulating MMA shows better stability compared to free Cb1 [14]. Circulating MMA shows better stability than Cb1, especially the free cobalamin. As cobalamin is a highly bound protein, the concentration of free cobalamin is difficult to reveal [14]. Also, the mass spectrometry method commonly used for MMA showed a higher specificity than the immunoassay commonly used for Cb1 [15, 16]. Therefore, increased concentrations of MMA can serve as a first-line functional indicator of Cb1 condition. Besides, the site of Hcy metabolism is widely distributed in the cytoplasm and its concentration is influenced by folic acid and vitamin B6, while in the mitochondria metabolism of MMA metabolism is directly determined by Cbl and mitochondrial MCM activity [17]. Although cellular damage due to Cb1 deficiency is partly attributed to the accumulation of Hcy, the concentration of circulating MMA has a higher sensitivity and specificity than Hcy to indicate the status of Cbl conditions. Compared to Hcy, MMA can be used as a first-line functional indicator of Cb1 viability. The relationship between MMA, Hcy, and Cb1 is presented in Figure 1.

### 2.2. MMA and Hereditary Methylmalonic Acidemia

Methylmalonic acidemia is an autosomal recessive disorder. Abnormal metabolism of the MMA cofactor 5-deoxyadenosyl cobalamin or defective MCM in the mitochondria results in the accumulation of large amounts of MMA in major tissues due to impaired metabolism [18, 19]. During acute episodes of methylmalonic acidemia, MMA accumulates in the blood and cerebrospinal fluid of patients [20, 21].

The metabolic blockage causes considerable MMA to be accumulated mainly in a tissue. Overall, concentrations of MMA in blood and cerebrospinal fluid are approximately 2.5 mmol/L during acute metabolic attacks [20, 21]. The catabolic metabolites of MMA (e.g., propionic, methyl citric and hydroxy propionic acids, and propionyl glycine) can also be detected in the patient's body fluids at the same time, but are not as easily detected as MMA due to its low concentration [22]. According to several available studies, MMA not only is a new risk factor for neurodegenerative diseases but also causes accumulation of organic acids and synergistic secondary toxic reactions [23], suggesting that acquired high levels of MMA can be a risk factor for adverse outcomes and not only an indicator of Cbl deficiency status.

Clinically, the major long-term complications consist of chronic renal failure [24] and neurological deficit [25], cardiomyopathy [26], pancreatitis [27], and recurrent infections attributed to leukopenia. Metabolic brain damage and the progression of heart disease can be induced [28]. Congenital methylmalonic acidemia adversely affects multiple organs, which may suggest the acquired high levels of MMA as a risk factor for adverse outcomes.

### 2.3. MMA and Cardiovascular Disease

Despite the lack of large-scale epidemiological studies on circulating MMA and coronary artery disease, MMA has been described as a risk factor for CHD in the available cross-sectional studies. The most frequent complications in the MMA group with renal disease are dilated cardiomyopathy and arterial hypertension [29]. Moreover, in a cross-sectional clinical study enrolled in a total of 120 patients, MMA serum levels significantly increased with acute myocardial infarction (AMI) or acute heart failure (HF) compared with healthy controls. This result suggested that the differences were independent of demographic, medical, and other comorbidities [6]. There were also studies in which patients with chronic decompensated HF had higher MMA concentrations than patients with newly diagnosed HF in the control group. A retrospective study also demonstrated that MMA levels in patients suffering from oxidative stress (e.g., atrial fibrillation or arterial hypertension) were elevated [30], since high levels of MMA may be related to cobalamin deficiency and impaired mitochondrial function, in addition to long-standing oxidative stress [31]. Accordingly, MMA critically impacts cardiac diseases, as the impairment of respiratory chain complex I have been identified in the cardiomyocytes, which inhibits carnitine uptake in the heart and causes cardiac insufficiency [32]. As suggested from a retrospective observational study in cblC-type methylmalonic aciduria, significant structural heart defects seem to be highly common probably due to MMA-influenced abnormal DNA methylation [33]. However, the mentioned studies have significant limitations, and convincing studies are rare on the association between MMA and the risk of cardiovascular events. Our recent cohort study in 23437 general adults demonstrated the significant relationship between circulating MMA and cardiovascular deaths [34]. Participants in MMA ≥ 250 nmol/L showed an increase in cardiovascular and all-cause mortality risk compared with those with MMA < 120 nmol/L. Thus, the accumulation of MMA is of critical importance for the evaluation of cardiovascular adverse events (risk and prognosis).

### 2.4. MMA and Other Chronic Diseases

It is known that plasma serum MMA levels increase above commonly accepted reference intervals with age [35]. Though vitamin B12 deficiency cannot be ruled out as a possibility contributing to the high level of MMA in the elderly, it may be related to other factors within the main organs [36]. Considerable data indicate a significant association between MMA and chronic diseases (e.g., renal dysfunction, neurodegenerative disease, obesity, and cancer) [2, 3].

To be specific, chronic renal failure is well-recognized complication of methylmalonic acidemia [24]. Moreover, the renal function acts as a vitally important determinant of MMA concentrations that is independent of vitamin B12 status in the patients [35]. The mitochondrial enrichment of epithelial cells of kidney tubules accounts for the transport functions and integrity [37]. The accumulation of MMA could break mitochondrial homeostasis and drive various degrees of tubular dysfunction [38]. As demonstrated by Horster and Hoffmann, accumulation of MMA on the tubular cell of the kidney could cause a disturbance of energy metabolism [39]. As opposed to the mentioned, kidney function might be restored by modulating mitochondrial function in mouse models [40]. In addition, tubular mitochondrial dysfunction refers to the key pathogenic mechanism of MMA-associated renal disease, while antioxidants were reported to reduce renal disease in some MMAs [41]. MMA can induce DNA damage in the kidney, which may explain kidney failure in patients of methylmalonic aciduria. Besides being toxic to the kidney, it is also known as a neurotoxin [42].

It is suggested that MMA, as an endogenous toxic metabolite, could impair energy metabolism [43, 44] and elicit oxidative stress in brain of rats [45]. It is demonstrated in a study that intrastriatal administration of MMA induces a change of behavior (e.g., rotational behavior and striatal lesions in rats) [46, 47]. MMA could induce neuron apoptosis in different cell culture systems and cause secondary excitotoxicity together with the complex II inhibitors malonate (MA) [48, 49]. As suggested from a longitudinal study in the United Kingdom, MMA is a significant predictor of cognitive impairment. The rate of decline in cognitive performance of subjects was upregulated by 50% with an increased concentration of MMA 0.25-0.50 *μ*mol/L in a longitudinal study in the United Kingdom [50]. The mentioned result might also explain the neurological deficit symptoms of methylmalonic acidemia which may have nonspecific symptoms (e.g., epilepsy or motor dysfunction of various degrees) [51–53]. These lesions typically occur during the acute phase of metabolic disorders. The neuroimaging of this inherited disease has shown basal ganglia degeneration and especially severe necrosis revealed by histopathology in the globus pallidus [4, 54]. By inhibiting the tricarboxylic acid cycle (TCA cycle) and mitochondrial respiratory chain, MMA causes one symptom of bioenergetic stroke after toxic metabolites accumulate [55].

According to one recent report, MMA could predict severe obesity together with homocysteine [56]. It is well known that insulin resistance is one of the key pathophysiological processes involved in obesity and diabetes mellitus. Some potential reasons might explain the Cb1 deficiency, and MMA could influence insulin resistance under the folate presence [57]. As a coenzyme, Cb1 could impair the activation efficiency of MMA and induce the expression of SIRT1 and lipogenesis subsequently [58, 59]. Studies have demonstrated that elevated MMA levels in diabetes patients showed more severe peripheral neuropathy [60, 61]. Similarly, our recent prospective cohort study in type 2 diabetes patients also found that MMA accumulation was positively associated with increased mortality risk [62]. Obesity and diabetes may play a critical biological role in the metabolic process of MMA in the setting of diseases.

Furthermore, MMA is a mediator of tumor progression by inducing aggressive features in cancer cells. As reported in a recent study, MMA is sufficient to stimulate the progression and aggressiveness of the tumor by inducing SOX4 by activating autocrine TGF*β* signaling. The accumulation of MMA in the aged host could represent antagonistic properties of cancer cells [36]. In brief, the association between MMA, an underestimated biomarker, and disease requires in-depth study and verification. As a systemically increased aging-induced metabolite [36], MMA could induce aggressive effects of aging in cancer cells and contribute to tumor progression and aggressiveness [63]. The pathophysiological mechanism related to MMA in the disease of cancer is not only mitochondrial dysfunction, impairment of tricarboxylic acid cycle, and oxidative stress mentioned before but also the effects of oncometabolites [36]. Several recent studies demonstrated that MMA could induce a proaggressive EMT-like phenotype with a decline in E-cadherin and a concurrent increase in fibronectin and vimentin. MMA is sufficient to endow cancer cells with migratory and invasive capacity by inducing SOX4 expression by activating autocrine TGF*β* signaling [35]. Therefore, MMA is indicated to be a potential therapeutic target in carcinoma treatment. In brief, the association between MMA, an underestimated biomarker, and disease requires in-depth study and verification.

## 3. Pathophysiology of MMA

### 3.1. Mitochondrial Homeostasis

Mitochondria are organelles with the energy of nutrients converted into adenosine triphosphate (ATP), which supports cellular metabolism and functions [64]. Thus, mitochondrial dysfunctions and homeostasis imbalances could result in crushing destruction to many cells, leading to a wide spectrum of diseases [65]. Accumulation of MMA due to mitochondrial dysfunction is recognized as the most common form of methylmalonic acidemia attributed to the mitochondrial enzyme MUT mutation and the lack of synthesis or transport of mitochondrial proteins [66, 67]. As a matter of fact, the metabolic pathway by which MMA enters the TCA cycle via propionyl-CoA and methylmalonyl-CoA produces large amounts of total ATP production under normal conditions [68]. In tissues and biological fluids, high levels of MMA might impair the energy metabolism of mitochondria. Disorders of mitochondrial energy metabolism consequently induce the elevation of intracellular free radical generation [5], leading to damage to mitochondrial DNA [69]. MMA is considered a mitochondrial toxin that interferes with redox equilibrium by inhibiting the electron transport complex II [4] and multiprotein in the TCA cycle, due to the exhibiting structural similarity with the respiratory chain complex II inhibitor MA [67]. Antagonists of ionotropic glutamate receptors and antioxidants prevented striatal lesions and cell injury induced by methyl methacrylate in rats [66]. Furthermore, one study suggests that MMA plays a role in inhibiting the transport of mitochondrial malate and succinate by a dicarboxylate carrier. Accordingly, one experiment demonstrated that MMA does not inhibit the consumption of succinate-supported oxygen in isolated mitochondria. Inhibition of the mitochondrial dicarboxylate carrier induced by methylmalonyl-CoA probably results in decreased gluconeogenesis and increased glycine in the kidneys and liver, and these could explain the disorders of failure to thrive and the delayed development in later childhood of methylmalonic acidurias [68, 70]. In the brain, the mitochondrial dicarboxylate carriers that could transport through the mitochondrial inner membrane are probably associated with de novo glutamate synthesis intermediates. Since pyruvate carboxylation is considered to occur only in astrocytes rather than neurons, high levels of MMA can compromise neuronal energy metabolism and glutamatergic neurotransmission [71]. In addition, MMA also inhibits the transport of glutathione in mitochondria via a dicarboxylate carrier at the same time inhibiting the mitochondrial dicarboxylate carrier, resulting in redox imbalance and mitochondrial antioxidant defense exhaustion [72]. As suggested by a number of studies, MMA leads to lipid peroxidation in cerebral tissues, which might explain the symptoms of neurologic deficit in methylmalonic acidemia [73–75].

Notably, MMA also shows a relationship to mitochondrial function and homeostasis. As discovered recently by Luciani et al., the MUT deficiency in methylmalonic acidemia might inhibit the autophagy of damaged mitochondria under stress-induced conditions by influencing Parkin's E3 ubiquitin ligase. Thus, damaged mitochondria may accumulate and generate epithelial stress and tissue injury [76]. MMA also induces mitochondrial damage via other mechanisms. In one study, the MMA metabolite was reported to suppress the activity of the citrate cycle rate-limiting enzyme, *α*-ketovalerate dehydrogenase complex (*α*KGDH), by competing with *α*-ketovalerate. The *α*KGDH activity was measured to decrease by 73% and 60% at high concentrations of MMA (10 mm) with 0.1 and 0.25 mm *α*-ketopentanoic acid, respectively. The mentioned effects will lead to a decrease in the number of intermediates in the TCA cycle, which can apparently damage the organs enriched with mitochondria by suppressing oxidative metabolism [28]. It has also been argued that MMA does not directly impact the mitochondrial respiratory chain. In addition, MMA-induced damage may be driven by metabolites derived from propionyl-CoA and its substitutes, including propionic, malonic, 2-methylcitric, and 3-hydroxypropionic acids, causing a synergistic inhibition of the TCA cycle and respiratory chain. As demonstrated by one study, the neuronal damage induced by MMA involves the intracellular accumulation of MA and 2-methylcitrate metabolite in rat embryos, thereby inhibiting the TAC in multiple pathways [55].

Mitochondria-rich organs in the body (e.g., heart, kidney, and brain) may also be affected by MMA to affect various functions [23]. It has been demonstrated in many studies that impaired mitochondrial function is closely related to cardiac ischemia-reperfusion injury [77, 78] and that improved mitochondrial quality control can reduce cardiac microvascular ischemia-reperfusion injury [79, 80]. As suggested by Wang et al. [81], MMA accumulation will result in significant trapping of mitochondrial coenzyme A in cardiomyocytes, promoting increased myocardial oxygen consumption and impeding normal cardiac productivity. Thus, circulating MMA is associated with heart failure and cardiac hypertrophy. On the other hand, MMA-induced mitochondrial damage also plays a pathogenic role in ischemic acute kidney injury (AKI) by disrupting mitochondrial mass and activating mitochondrial apoptosis [82, 83]. However, few relevant in vivo studies have been conducted on the biological function of methyl methacrylate in cardiovascular disorders, and the potential clinical significance of MMA remains unclear.

### 3.2. Oxidative Stress

MMA, as a promising novel biomarker, may represent the condition of oxidative stress [6]. Oxidative stress is identified as an important contributor to physiopathology of several diseases including cancer [84] and metabolic diseases [85]. There have been numerous studies based on animal models, and patients report the existence of oxidative stress within methylmalonic acidemia [86–88]. One experiment demonstrated that primary neuronal cultures and mouse models have suffered by significant toxic effects by consecutive intrastriatal administration [66]. And another laboratory reported that injecting MMA into the encephalocoele in animal models could interfere with redox homeostasis [88]. The source of oxidative stress is usually multifactorial and seldom attributable to a single mechanism [89]. These factors include the accumulation of toxic metabolites in metabolic diseases and the production of reactive oxygen species (ROS) as well as reactive nitrogen species (RNS) related to pathogenesis of other diseases. In methylmalonic acidemia, the primary reason for oxidative stress is considered to be the generation of mitochondrial ROS influenced by electron transport chain (ETC) dysfunction [73]. The results of some studies have suggested that inhibiting the enzymatic activity of ETC due to the accumulation of malonate and methylcitrate rather than MMA itself [55]. However, the results from other studies indicate that MMA tends to inhibit ETC activity [90–92]. Accordingly, synergistic inhibition by MMA, methylcitrate, and malonate might be responsible for the ETC dysfunction associated with methylmalonic acidemia [21].

Oxidative stress inevitably results in oxidative damage of proteins and lipids as well as a decrease in the antioxidant defense in vivo, while succinic acid, antagonists of ionotropic glutamate receptors, and antioxidants were prone to effectively prevent injury induced by MMA owing to their antioxidant [66]. There is extensive evidence that the antioxidant status of cells has an impact on methylmalonic acidemia. However, few studies have suggested antioxidant as an adjunct therapy to the methylmalonic acidemia treatment regimen. According to an animal model of methylmalonic acidemia, the combination of CoQ10 and vitamin E improves the glomerular filtration rate [41]. Furthermore, Salmi et al. showed that patients with methylmalonic acidemia have a deficiency of glutathione and have an overproduction of Oxic-nitric (NO) [93]. There is also evidence that protein damage is mediated by NO, since seizures induced by MMA decline significantly in endothelial nitric oxide synthase knockout mice compared to normal controls [68, 94]. Thus, the increasing dose of MMA is also suggested to be able to reduce immune defenses. These findings may have the potential to offer a novel biomarker for disease prevention and treatment.

MMA along with Hcy serum levels are significantly elevated at the beginning of vitamin B12 deficiency, so both can be adopted to detect the vitamin B12 deficiency condition. Under normal conditions, MMA participates in the TCA cycle that requires Cb1 in the formation of adenosylcobalamin (AdoCbl) to be a cofactor of this chemical reaction [95]. Additionally, Cb1 is involved in converting Hcy into methionine and leads to methyl group generation through the tetrahydrofolate cycle [96]. Hcy has been extensively reported as a critical risk factor for the cardiovascular system and neurodegenerative diseases [97, 98]. Since existing studies suggested a positive relationship between Hcy and the severity of coronary heart disease, it plays a predictive role for guiding the disease assessment of coronary heart disease [16, 99]. Moreover, several studies reported that Hcy can activate nicotinamide adenine dinucleotide phosphate (NADPH) oxidase and generate massive production of ROS that causes damage to vascular endothelial cells and promotes lipid peroxidation and oxidation of low-density lipoproteins. Hcy could enhance oxidative activity and aggravate cellular oxidative stress injury [100, 101], thereby causing vascular damage and progression of atherosclerotic plaque to be aggravated. Though cell damage for B12 deficiency is partially attributed to accumulation of Hcy, the concentration of circulating MMA has more sensitivity and specificity to indicate the state of Cbl condition than for Hcy [8]. The site of Hcy metabolism is extensively cytoplasmic. However, MMA metabolism is directly determined by Cbl and mitochondrial MCM activity; it is not dependent of folic acid and vitamin B6 [17]. Figure 1 lists the relationship between MMA, Hcy, and Cb1. Thus, MMA may reflect oxidative stress-related pathological impairment than high homocysteine as a biomarker.

### 3.3. Neuronal Cell Apoptosis

Neuronal cell apoptosis may be one of the mechanisms related to the progression of MMA-induced disease. In a number of studies, MMA causes a decreased intracellular ATP/ADP ratio and depolarization of the plasma membrane in cultured neurons, eventually resulting in necrotic and apoptotic cell death [102]. Besides, high levels of MMA probably cause the interference of MAPK and p53 signaling pathways to decrease neuron viability and increase cell apoptosis [103]. Ionotropic glutamate antagonists' receptors could be used to prevent MMA-induced cell death, which suggests that excitotoxic mechanisms are involved in this pathology of cellular damage [66]. Okun et al. reported that MMA loading in rats led to intracellular accumulation of 2-methylcitric acid (2-MCA) and MA induce cellular damage [66]. For this reason, the induction of MMA may be indirect, which involves MMA and MA acting synergistically to mediate the impairment of cellular energy metabolism [55]. The release of glutamate, which is mainly expressed by the overactivation of N-methyl-D-aspartate (NMDA) receptors and induces an influx of Ca^2+^ and Na^+^ subsequently, could relate to the process of central nervous system [104]. Under excitotoxicity conditions, high doses of stressors, such as the mitochondrial matrix Ca2+ and ROS, may cause rupture of the outer mitochondrial membrane and mitochondrial dysfunction through mitochondrial permeability transition (MPT) [105]. As suggested by Kowaltowski et al., MPT was involved in MMA-mediated neurotoxicity, since cyclosporin A (an MPT inhibitor) has been found to prevent MMA-induced cell death [102]. Furthermore, increasing evidences have suggested that the pathogenesis of MMA is related to the dysfunction of intracellular trafficking [106]. These can explain the symptoms of neurologic deficiency in methylmalonic acidemia.

## 4. Summary

It is acknowledged that MMA is capable of monitoring early vitamin B12 deficiency and diagnosing genetic metabolic disorders clinically. Moreover, the metabolism of MMA depends on mitochondrial status, and MMA also affects the energy homeostasis of mitochondria. MMA metabolism also affects the deterioration of diseases characterized by mitochondrial impairment, including cardiovascular disease, chronic renal failure, neurodegenerative disease, overweight, and cancer. Accordingly, MMA might show a substantial potential to improve disease management and risk stratification by complying with its distinctive biological role. There has been insufficient evidence on the relationship between MMA and a series of diseases and its prognostic value. A considerable number of studies face obvious limitations (e.g., small sample size, insufficient sensitivity of detection methods, and inconsistent diagnostic criteria). MMA in the pathogenesis and clinical risk stratification in mitochondrial-related disease warrants further elucidation.

## Figures and Tables

**Figure 1:** The relationship between MMA, Hcy, and Cb1.

## References

[1] Cox E. V., White A. M. (1962). Methylmalonic acid excretion: an index of vitamin-B_12_ deficiency. *Lancet*.

[2] Mineva E. M., Sternberg M. R., Zhang M. (2019). Age-specific reference ranges are needed to interpret serum methylmalonic acid concentrations in the US population. *The American Journal of Clinical Nutrition*.

[3] Liu X., Gao X., Zhang R. (2020). Discovery and comparison of serum biomarkers for diabetes mellitus and metabolic syndrome based on UPLC-Q-TOF/MS. *Clinical Biochemistry*.

[4] Larnaout A., Mongalgi M. A., Kaabachi N. (1998). Methylmalonic acidaemia with bilateral globus pallidus involvement: a neuropathological study. *Journal of Inherited Metabolic Disease*.

[5] Indo H. P., Davidson M., Yen H. C. (2007). Evidence of ROS generation by mitochondria in cells with impaired electron transport chain and mitochondrial DNA damage. *Mitochondrion*.

[6] Polytarchou K., Dimitroglou Y., Varvarousis D. (2020). Methylmalonic acid and vitamin B12 in patients with heart failure. *Hellenic Journal of Cardiology*.

[7] Elin R. J., Winter W. E. (2001). Methylmalonic acid. *Archives of Pathology & Laboratory Medicine*.

[8] Hannibal L., Lysne V., Bjørke-Monsen A. L., Behringer S., Grünert S. C., Spiekerkoetter U. (2016). Biomarkers and algorithms for the diagnosis of vitamin B12 deficiency. *Frontiers in Molecular Biosciences*.

[9] Suormala T., Baumgartner M. R., Coelho D. (2004). The cblD defect causes either isolated or combined deficiency of methylcobalamin and adenosylcobalamin synthesis. *The Journal of Biological Chemistry*.

[10] Obeid R., Jung J., Falk J. (2013). Serum vitamin B12 not reflecting vitamin B12 status in patients with type 2 diabetes. *Biochimie*.

[11] Vashi P., Edwin P., Popiel B., Lammersfeld C., Gupta D. (2016). Methylmalonic acid and homocysteine as indicators of vitamin B-12 deficiency in cancer. *PLoS One*.

[12] Bailey R. L., Carmel R., Green R. (2011). Monitoring of vitamin B-12 nutritional status in the United States by using plasma methylmalonic acid and serum vitamin B-12. *The American Journal of Clinical Nutrition*.

[13] Yao Y., Yao S. L., Yao S. S., Yao G., Lou W. (1992). Prevalence of vitamin B12 deficiency among geriatric outpatients. *The Journal of Family Practice*.

[14] Wickramasinghe S. N., Fida S. (1993). Correlations between holo-transcobalamin II, holo-haptocorrin, and total B12 in serum samples from healthy subjects and patients. *Journal of Clinical Pathology*.

[15] Clarke R., Refsum H., Birks J. (2003). Screening for vitamin B-12 and folate deficiency in older persons. *The American Journal of Clinical Nutrition*.

[16] Biselli P. M., Guerzoni A. R., de Godoy M. F. (2010). Genetic polymorphisms involved in folate metabolism and concentrations of methylmalonic acid and folate on plasma homocysteine and risk of coronary artery disease. *Journal of Thrombosis and Thrombolysis*.

[17] Aarsetoy H., Valente E., Reine A., Mansoor M. A., Grundt H., Nilsen D. W. T. (2008). Holotranscobalamin and methylmalonic acid as prognostic markers following an acute myocardial infarction. *European Journal of Clinical Nutrition*.

[18] Baumgartner M. R., Hörster F., Dionisi-Vici C. (2014). Proposed guidelines for the diagnosis and management of methylmalonic and propionic acidemia. *Orphanet Journal of Rare Diseases*.

[19] Chandler R. J., Venditti C. P. (2019). Gene therapy for methylmalonic acidemia: past, present, and future. *Human Gene Therapy*.

[20] Imperlini E., Santorelli L., Orrù S., Scolamiero E., Ruoppolo M., Caterino M. (2016). Mass spectrometry-based metabolomic and proteomic strategies in organic acidemias. *BioMed Research International*.

[21] Treacy E., Arbour L., Chessex P. (1996). Glutathione deficiency as a complication of methylmalonic acidemia: response to high doses of ascorbate. *The Journal of Pediatrics*.

[22] van der Meer S. B., Poggi F., Spada M. (1994). Clinical outcome of long-term management of patients with vitamin B_12_-unresponsive methylmalonic acidemia. *The Journal of Pediatrics*.

[23] Ganji V., Kafai M. R. (2012). Population prevalence, attributable risk, and attributable risk percentage for high methylmalonic acid concentrations in the post-folic acid fortification period in the US. *Nutrition & Metabolism (London)*.

[24] Baumgarter E. R., Viardot C., 147 colleagues of 39 hospitals from 7 European countries (1995). Long-term follow-up of 77 patients with isolated methylmalonic acidaemia. *Journal of Inherited Metabolic Disease*.

[25] Nicolaides P., Leonard J., Surtees R. (1998). Neurological outcome of methylmalonic acidaemia. *Archives of Disease in Childhood*.

[26] Massoud A. F., Leonard J. V. (1993). Cardiomyopathy in propionic acidaemia. *European Journal of Pediatrics*.

[27] Kahler S. G., Sherwood W. G., Woolf D. (1994). Pancreatitis in patients with organic acidemias. *The Journal of Pediatrics*.

[28] Morath M. A., Okun J. G., Müller I. B. (2008). Neurodegeneration and chronic renal failure in methylmalonic aciduria—a pathophysiological approach. *Journal of Inherited Metabolic Disease*.

[29] Kolker S., Valayannopoulos V., Burlina A. B. (2015). The phenotypic spectrum of organic acidurias and urea cycle disorders. Part 2: the evolving clinical phenotype. *Journal of Inherited Metabolic Disease*.

[30] Solomon L. R. (2016). Low cobalamin levels as predictors of cobalamin deficiency: importance of comorbidities associated with increased oxidative stress. *The American Journal of Medicine*.

[31] Solomon L. R. (2015). Functional cobalamin (vitamin B12) deficiency: role of advanced age and disorders associated with increased oxidative stress. *European Journal of Clinical Nutrition*.

[32] Ou P., Touati G., Fraisse A. (2001). A rare cause of cardiomyopathy in childhood: propionic acidosis. Three case reports. *Archives des Maladies du Coeur et des Vaisseaux*.

[33] Profitlich L. E., Kirmse B., Wasserstein M. P., Diaz G. A., Srivastava S. (2009). High prevalence of structural heart disease in children with cblC-type methylmalonic aciduria and homocystinuria. *Molecular Genetics and Metabolism*.

[34] Wang S., Liu Y., Liu J. (2020). Mitochondria-derived methylmalonic acid, a surrogate biomarker of mitochondrial dysfunction and oxidative stress, predicts all-cause and cardiovascular mortality in the general population. *Redox Biology*.

[35] Lewerin C., Ljungman S., Nilsson-Ehle H. (2007). Glomerular filtration rate as measured by serum cystatin C is an important determinant of plasma homocysteine and serum methylmalonic acid in the elderly. *Journal of Internal Medicine*.

[36] Gomes A. P., Ilter D., Low V. (2020). Age-induced accumulation of methylmalonic acid promotes tumour progression. *Nature*.

[37] Forbes J. M. (2016). Mitochondria-power players in kidney function?. *Trends in Endocrinology and Metabolism*.

[38] Emma F., Montini G., Parikh S. M., Salviati L. (2016). Mitochondrial dysfunction in inherited renal disease and acute kidney injury. *Nature Reviews. Nephrology*.

[39] Horster F., Hoffmann G. F. (2004). Pathophysiology, diagnosis, and treatment of methylmalonic aciduria-recent advances and new challenges. *Pediatric Nephrology*.

[40] Jesinkey S. R., Funk J. A., Stallons L. J. (2014). Formoterol restores mitochondrial and renal function after ischemia-reperfusion injury. *J Am Soc Nephrol*.

[41] Manoli I., Sysol J. R., Li L. (2013). Targeting proximal tubule mitochondrial dysfunction attenuates the renal disease of methylmalonic acidemia. *Proceedings of the National Academy of Sciences of the United States of America*.

[42] Andrade V. M., Dal Pont H. S., Leffa D. D. (2014). Methylmalonic acid administration induces DNA damage in rat brain and kidney. *Molecular and Cellular Biochemistry*.

[43] Schuck P. F., Rosa R. B., Pettenuzzo L. F. (2004). Inhibition of mitochondrial creatine kinase activity from rat cerebral cortex by methylmalonic acid. *Neurochemistry International*.

[44] Pettenuzzo L. F., Ferreira G. . C., Schmidt A. L., Dutra-Filho C. S., Wyse A. T. S., Wajner M. (2006). Differential inhibitory effects of methylmalonic acid on respiratory chain complex activities in rat tissues. *International Journal of Developmental Neuroscience*.

[45] Pettenuzzo L. F., Schuck P.´. F., Wyse A. T. S. (2003). Ascorbic acid prevents water maze behavioral deficits caused by early postnatal methylmalonic acid administration in the rat. *Brain Research*.

[46] de Mello C. F., Begnini J., Jiménez-Bernal R. E. (1996). Intrastriatal methylmalonic acid administration induces rotational behavior and convulsions through glutamatergic mechanisms. *Brain Research*.

[47] Narasimhan P., Sklar R., Murrell M., Swanson R. A., Sharp F. R. (1996). Methylmalonyl-CoA mutase induction by cerebral ischemia and neurotoxicity of the mitochondrial toxin methylmalonic acid. *The Journal of Neuroscience*.

[48] Kolker S., Ahlemeyer B., Krieglstein J., Hoffmann G. F. (2000). Methylmalonic acid induces excitotoxic neuronal damage in vitro. *Journal of Inherited Metabolic Disease*.

[49] Beal M. F., Brouillet E., Jenkins B. G. (1993). Neurochemical and histologic characterization of striatal excitotoxic lesions produced by the mitochondrial toxin 3-nitropropionic acid. *The Journal of Neuroscience*.

[50] Clarke R., Birks J., Nexo E. (2007). Low vitamin B-12 status and risk of cognitive decline in older adults. *The American Journal of Clinical Nutrition*.

[51] Surtees R. A., Matthews E. E., Leonard J. V. (1992). Neurologic outcome of propionic acidemia. *Pediatric Neurology*.

[52] Shevell M. I., Matiaszuk N., Ledley F. D., Rosenblatt D. S. (1993). Varying neurological phenotypes among mut° and mut− patients with methylmalonylCoA mutase deficiency. *American Journal of Medical Genetics*.

[53] de Baulny H. O., Benoist J. F., Rigal O., Touati G., Rabier D., Saudubray J. M. (2005). Methylmalonic and propionic acidaemias: management and outcome. *Journal of Inherited Metabolic Disease*.

[54] Brismar J., Ozand P. T. (1994). CT and MR of the brain in disorders of the propionate and methylmalonate metabolism. *AJNR. American Journal of Neuroradiology*.

[55] Kolker S., Schwab M., Horster F. (2003). Methylmalonic acid, a biochemical hallmark of methylmalonic acidurias but no inhibitor of mitochondrial respiratory chain. *The Journal of Biological Chemistry*.

[56] Li Z., Gueant-Rodriguez R. M., Quilliot D. (2018). Folate and vitamin B12 status is associated with insulin resistance and metabolic syndrome in morbid obesity. *Clinical Nutrition*.

[57] Selhub J., Rosenberg I. H. (2016). Excessive folic acid intake and relation to adverse health outcome. *Biochimie*.

[58] Krishnaveni G. V., Hill J. C., Veena S. R. (2009). Low plasma vitamin B12 in pregnancy is associated with gestational 'diabesity' and later diabetes. *Diabetologia*.

[59] Krishnaveni G. V., Hill J. C., Leary S. D. (2005). Anthropometry, glucose tolerance, and insulin concentrations in Indian children: relationships to maternal glucose and insulin concentrations during pregnancy. *Diabetes Care*.

[60] Wile D. J., Toth C. (2010). Association of metformin, elevated homocysteine, and methylmalonic acid levels and clinically worsened diabetic peripheral neuropathy. *Diabetes Care*.

[61] Sun A. L., Ni Y.-h., Li X.-b. (2014). Urinary methylmalonic acid as an indicator of early vitamin B12 deficiency and its role in polyneuropathy in type 2 diabetes. *Journal Diabetes Research*.

[62] Wang S., Wang Y., Wan X. (2022). Cobalamin intake and related biomarkers: examining associations with mortality risk among adults with type 2 diabetes in NHANES. *Diabetes Care*.

[63] Gomes A. P., Ilter D., Low V. (2022). Altered propionate metabolism contributes to tumour progression and aggressiveness. *Nature Metabolism*.

[64] Nunnari J., Suomalainen A. (2012). Mitochondria: in sickness and in health. *Cell*.

[65] Johannsen D. L., Ravussin E. (2009). The role of mitochondria in health and disease. *Current Opinion in Pharmacology*.

[66] Okun J. G., Hörster F., Farkas L. M. (2002). Neurodegeneration in methylmalonic aciduria involves inhibition of complex II and the tricarboxylic acid cycle, and synergistically acting excitotoxicity. *The Journal of Biological Chemistry*.

[67] Wajner M., Coelho J. C. (1997). Neurological dysfunction in methylmalonic acidaemia is probably related to the inhibitory effect of methylmalonate on brain energy production. *Journal of Inherited Metabolic Disease*.

[68] Villani G. R., Gallo G., Scolamiero E., Salvatore F., Ruoppolo M. (2017). "Classical organic acidurias": diagnosis and pathogenesis. *Clinical and Experimental Medicine*.

[69] Wallace D. C. (2005). The mitochondrial genome in human adaptive radiation and disease: on the road to therapeutics and performance enhancement. *Gene*.

[70] Mirandola S. R., Melo D. R., Schuck P. F., Ferreira G. C., Wajner M., Castilho R. F. (2008). Methylmalonate inhibits succinate-supported oxygen consumption by interfering with mitochondrial succinate uptake. *Journal of Inherited Metabolic Disease*.

[71] Sheng S., Moraga-Amador D. A., van Heeke G., Allison R. D., Richards N. G., Schuster S. M. (1993). Glutamine inhibits the ammonia-dependent activities of two Cys-1 mutants of human asparagine synthetase through the formation of an abortive complex. *The Journal of Biological Chemistry*.

[72] Lash L. H. (2006). Mitochondrial glutathione transport: physiological, pathological and toxicological implications. *Chemico-Biological Interactions*.

[73] Fontella F. U., Pulrolnik V., Gassen E. (2000). Propionic and L-methylmalonic acids induce oxidative stress in brain of young rats. *Neuroreport*.

[74] Malfatti C. R., Royes L. F. F., Francescato L. (2003). Intrastriatal methylmalonic acid administration induces convulsions and TBARS production, and alters Na+,K+-ATPase activity in the rat striatum and cerebral cortex. *Epilepsia*.

[75] Maciel E. N., Kowaltowski A. J., Schwalm F. D. (2004). Mitochondrial permeability transition in neuronal damage promoted by Ca^2+^ and respiratory chain complex II inhibition. *Journal of Neurochemistry*.

[76] Luciani A., Schumann A., Berquez M. (2020). Impaired mitophagy links mitochondrial disease to epithelial stress in methylmalonyl-CoA mutase deficiency. *Nature Communications*.

[77] Zhou H., Toan S., Zhu P., Wang J., Ren J., Zhang Y. (2020). DNA-PKcs promotes cardiac ischemia reperfusion injury through mitigating BI-1-governed mitochondrial homeostasis. *Basic Research in Cardiology*.

[78] Wang J., Toan S., Zhou H. (2020). New insights into the role of mitochondria in cardiac microvascular ischemia/reperfusion injury. *Angiogenesis*.

[79] Wang J., Zhou H. (2020). Mitochondrial quality control mechanisms as molecular targets in cardiac ischemia – reperfusion injury. *Acta Pharmaceutica Sinica B*.

[80] Tan Y., Mui D., Toan S., Zhu P., Li R., Zhou H. (2020). SERCA overexpression improves mitochondrial quality control and attenuates cardiac microvascular ischemia-reperfusion injury. *Mol Ther Nucleic Acids*.

[81] Wang Y., Christopher B. A., Wilson K. A. (2018). Propionate-induced changes in cardiac metabolism, notably CoA trapping, are not altered by l-carnitine. *American Journal of Physiology. Endocrinology and Metabolism*.

[82] Chen R. (2020). Guideline on therapeutic use of repetitive transcranial magnetic stimulation: useful but know the methods and limitations. *Clinical Neurophysiology*.

[83] Wang J., Zhu P., Li R., Ren J., Zhang Y., Zhou H. (2020). Bax inhibitor 1 preserves mitochondrial homeostasis in acute kidney injury through promoting mitochondrial retention of PHB2. *Theranostics*.

[84] Sosa V., Moliné T., Somoza R., Paciucci R., Kondoh H., LLeonart M. E. (2013). Oxidative stress and cancer: an overview. *Ageing Research Reviews*.

[85] van Bakel M. M., Printzen G., Wermuth B., Wiesmann U. N. (2000). Antioxidant and thyroid hormone status in selenium-deficient phenylketonuric and hyperphenylalaninemic patients. *The American Journal of Clinical Nutrition*.

[86] Ribas G. S., Sitta A., Wajner M., Vargas C. R. (2011). Oxidative stress in phenylketonuria: what is the evidence?. *Cellular and Molecular Neurobiology*.

[87] Atkuri K. R., Cowan T. M., Kwan T. (2009). Inherited disorders affecting mitochondrial function are associated with glutathione deficiency and hypocitrullinemia. *Proceedings of the National Academy of Sciences of the United States of America*.

[88] Viegas C. M., Zanatta Â., Grings M. (2014). Disruption of redox homeostasis and brain damage caused in vivo by methylmalonic acid and ammonia in cerebral cortex and striatum of developing rats. *Free Radical Research*.

[89] Stepien K. M., Heaton R., Rankin S. (2017). Evidence of oxidative stress and secondary mitochondrial dysfunction in metabolic and non-metabolic disorders. *Journal of Clinical Medicine*.

[90] Brusque A. M., Borba Rosa R., Schuck P. F. (2002). Inhibition of the mitochondrial respiratory chain complex activities in rat cerebral cortex by methylmalonic acid. *Neurochemistry International*.

[91] Royes L. F., Fighera M. R., Furian A. F. (2003). Creatine protects against the convulsive behavior and lactate production elicited by the intrastriatal injection of methylmalonate. *Neuroscience*.

[92] Fleck J., Ribeiro M. C. P., Schneider C. M., Sinhorin V. D. G., Rubin M. A., Mello C. F. (2004). Intrastriatal malonate administration induces convulsive behaviour in rats. *Journal of Inherited Metabolic Disease*.

[93] Salmi H., Leonard J. V., Lapatto R. (2012). Patients with organic acidaemias have an altered thiol status. *Acta Paediatrica*.

[94] Ribeiro L. R., Della-Pace I. D., de Oliveira Ferreira A. P. (2013). Chronic administration of methylmalonate on young rats alters neuroinflammatory markers and spatial memory. *Immunobiology*.

[95] Green R., Allen L. H., Bjørke-Monsen A. L. (2017). Vitamin B_12_ deficiency. *Nature Reviews. Disease Primers*.

[96] Finkelstein J. D., Martin J. J. (2000). Homocysteine. *The International Journal of Biochemistry & Cell Biology*.

[97] Veeranna V., Zalawadiya S. K., Niraj A. (2011). Homocysteine and reclassification of cardiovascular disease risk. *Journal of the American College of Cardiology*.

[98] Hannibal L., Blom H. J. (2017). Homocysteine and disease: causal associations or epiphenomenons?. *Molecular Aspects of Medicine*.

[99] Glueck C. J., Shaw P., Lang J. E., Tracy T., Sieve-Smith L., Wang Y. (1995). Evidence that homocysteine is an independent risk factor for atherosclerosis in hyperlipidemic patients. *The American Journal of Cardiology*.

[100] van de Lagemaat E. E., de Groot L., van den Heuvel E. G. (2019). Vitamin B12 in relation to oxidative stress: a systematic review. *Nutrients*.

[101] Bito T., Misaki T., Yabuta Y., Ishikawa T., Kawano T., Watanabe F. (2017). Vitamin B_12_ deficiency results in severe oxidative stress, leading to memory retention impairment in _Caenorhabditis elegans_. *Redox Biology*.

[102] Kowaltowski A. J., Maciel E. N., Fornazari M., Castilho R. F. (2006). Diazoxide protects against methylmalonate-induced neuronal toxicity. *Experimental Neurology*.

[103] Han L., Wu S., Han F., Gu X. (2015). Insights into the molecular mechanisms of methylmalonic acidemia using microarray technology. *International Journal of Clinical and Experimental Medicine*.

[104] Nicholls D. G., Budd S. L. (2000). Mitochondria and neuronal survival. *Physiological Reviews*.

[105] Kowaltowski A. J., Seetharaman S., Paucek P., Garlid K. D. (2001). Bioenergetic consequences of opening the ATP-sensitive K(+) channel of heart mitochondria. *American Journal of Physiology. Heart and Circulatory Physiology*.

[106] De Mattos-Dutra A., De Freitas M. S., Schröder N., Zilles A. C., Wajner M., Pessoa-Pureur R. (1997). Methylmalonic acid reduces the in vitro phosphorylation of cytoskeletal proteins in the cerebral cortex of rats. *Brain Research*.

